# Gauging the Impact of Artificial Intelligence and Mathematical Modeling in Response to the COVID-19 Pandemic: A Systematic Review

**DOI:** 10.1155/2022/7731618

**Published:** 2022-03-14

**Authors:** Afshan Hassan, Devendra Prasad, Shalli Rani, Musah Alhassan

**Affiliations:** ^1^Chitkara University Institute of Engineering and Technology, Chitkara University, Punjab, India; ^2^University of Development Studies, Electrical Engineering Department, School of Engineering, Nyankpala Campus, Ghana

## Abstract

While the world continues to grapple with the devastating effects of the SARS-nCoV-2 virus, different scientific groups, including researchers from different parts of the world, are trying to collaborate to discover solutions to prevent the spread of the COVID-19 virus permanently. Henceforth, the current study envisions the analysis of predictive models that employ machine learning techniques and mathematical modeling to mitigate the spread of COVID-19. A systematic literature review (SLR) has been conducted, wherein a search into different databases, viz., PubMed and IEEE Explore, fetched 1178 records initially. From an initial of 1178 records, only 50 articles were analyzed completely. Around (64%) of the studies employed data-driven mathematical models, whereas only (26%) used machine learning models. Hybrid and ARIMA models constituted about (5%) and (3%) of the selected articles. Various Quality Evaluation Metrics (QEM), including accuracy, precision, specificity, sensitivity, Brier-score, F1-score, RMSE, AUC, and prediction and validation cohort, were used to gauge the effectiveness of the studied models. The study also considered the impact of Pfizer-BioNTech (BNT162b2), AstraZeneca (ChAd0x1), and Moderna (mRNA-1273) on Beta (B.1.1.7) and Delta (B.1.617.2) viral variants and the impact of administering booster doses given the evolution of viral variants of the virus.

## 1. Introduction

Since the 29th of December, 2019, the epidemic of a new coronavirus broke out starting from China that created havoc and dismay all over the world [1]. Coronavirus belongs to a family of viruses with positive-sense (+) RNA (ribonucleic acid), which have the capability of infecting the host by inducing the host with symptoms of cold and flu in its mild stage and severe respiratory ailments and multiorgan failure in its lethal stage [2]. This virus can infect humans, and several cases of pets getting infected (Figure 1) have also been reported in different parts of the world. Some countries have a history of underreporting the disease, and it acts as a catalyst in the spread of infection. Lack of infrastructure, proper testing techniques, and high population may be the reasons for the spread of this deadly virus throughout the countries, continents, and subcontinents [3]. Various countries like China, Japan, and Singapore, which reported a higher number of cases initially in the first stage of the virus, have managed to slow down the rate of infection compared to countries like India and the U.S. [4]. The positive COVID-19 cases in India continue to rise; however, the lockdown, social distancing, and other measures have been implemented, and the measurable effect is yet to take place on a more significant note [5].

This global pandemic has severe implications on people's health and negatively impacts businesses and the economy. On average, the cumulative cases of COVID-19 are increasing day by day; although, some countries like Canada, Taiwan, and Iceland have succeeded in flattening the curve [6]. However, with the global race for vaccine intensifying and theories about plasma technology and herd immunity coming to the surface, the apprehensions about its intensification seem to subside. Still, for some, it raises eyebrows [7]. Moreover, there is little knowledge of what challenges could arise during the development, which could further delay the timelines.

The spread of this newly emerging virus still holds uncertainty regarding current and future behavior; although, numerous studies suggesting that the trend worldwide have been reported. The role of the airline travel network seems to be pivotal in the spreading of COVID-19, which has led to the development of several mathematical modeling techniques that enable us to examine the present status and demonstrate the future predictions of any eventuality [8]. In addition, numerous researchers have studied the number of confirmed, recovered, and death cases within a specific time frame for various countries to identify the various stages in the plots among different states under study [9]. The possible outcomes in many studies show a positive relationship between global transportation networks and the spread of the disease [10].

The disease can transmit either horizontally or vertically within the population. Horizontal transmission occurs through direct or indirect contact with infected individuals, whereas vertical transmission involves the transmission of diseases from mother to unborn offspring [11]. The implementation of lockdown and quarantine, restrictions implemented on social gatherings, somehow has provided some sort of relaxations and hence enough time for healthcare systems to prepare for the inevitable. Still, it seems pretty harsh to implement unprecedented stringent preventive measures to mitigate or contain the infection in different setups [12].

The lack of efficacy for creating awareness among the masses, absence of effective measures, and medical equipment to ensure public health safety in the early stages of the spread of this virus led to its uncontrollable breakout. Several predictive models proposed so far for understanding the trend of COVID-19 employ variable datasets and deduce many disease-related parameters [13]. These models claim to hold the imprimatur of the science of COVID-19 disease transmission. Given the highly mutating nature of the virus, there is a risk that a more virulent or more transmissible mutation of the COVID-19 strain may crop up, resulting in the successive waves of COVID-19. This necessitates the study and deployment of appropriate surveillance and containment measures to contain the consecutive waves of the COVID-19 pandemic [14]. Therefore, an SLR study is a must to identify and understand the effective machine learning and mathematical models employed for mitigating the spread of COVID-19 while summarizing and marking the effective solutions from the identified literature.  Section 2 epitomizes the background and motivation of the study. The methodology employed for performing systematic literature review (SLR) on the spread of COVID-19 is outlined in Section 3.  Section 4 confers to the results and discussions on the identified research questions. The limitations of this study are addressed in Section 5.

## 2. Background and Motivation

### 2.1. Progression of Successive Waves of COVID-19 and the Evolution of Viral Variants

On average, the global count of confirmed cases of COVID-19 has crossed the mark of 271 million, with more than 7 million deaths reported worldwide up to 13^th^ December 2021. With the global race for vaccine intensifying, China is administering almost more than 2.6 billion and 1.3 billion doses of vaccine. India and the U.S. follow this (see Figure 2). However, there is still a concern about the successive waves of.

COVID-19 hitting the different parts of the world attributed to the evolution of viral variants of the COVID-19 virus. Starting from February 2020 till Oct 2021, Asia was the center of infections emerging from Wuhan, China, in early 2019. More than 22 million cases were recorded in Brazil, with 617,000 deaths, the highest during the aforementioned period. Recently, many European countries, including Russia, Ukraine, Germany, and Poland, saw a sudden surge in COVID-19 infections, driven by the Delta variant of the COVID-19 virus, in early June 2021. The World Health Organization (WHO) has declared Europe as the epicenter of the pandemic, with the U.K. reporting the highest number of COVID-19 infections. The U.S. has reported around 50 million cases with 800,000 deaths globally. In response to the Omicron variant [15], North American countries have incorporated travel restrictions and updated vaccination status (see Figure 3). Several countries in the Middle East have seen severe outbreaks of the virus. The death toll for Iran is more than 1,30,000. Intending to keep the daily infections due to the Omicron variant under check, many countries have given booster shots to their population [16]. According to the official figures, South Africa is the worst affected continent with more than 3 million COVID-19 cases and around 1 lakh death.

In order to enhance the collaboration and coordination among the National Institute of Health (NIH) and the Department of Defence (DoD), a SARS-COVID-19 Interagency Group (SIG) was established by the Health Department of the U.S. [18]. The aim was the monitoring of emerging variants and their impact on the countermeasures viz., vaccines and therapeutics, to align with the aforementioned for well-preparedness against COVID-19 infection. World Health Organization (WHO) categorizes the evolving COVID-19 mutants into three groups, [19] viz., variants of interest, variants of concern, and variants of high consequence as in Table 1.

#### 2.1.1. Variants of Interest (VOI)

These variants of SARS-COVID-19 are characterized by changes in transmissibility or virulence of COVID-19 infection, with a probable increase in the infection rates and a partial neutralizing effect on the antibodies developed because of prior infection or through vaccination.

#### 2.1.2. Variants of Concern (VOC)

These variants are characterized by the following:

- All attributes of VOI
- Evidence of markers capable of increasing the infection or death rates
- There is evidence of neutralizing effect on antibodies, prevention, therapeutics, or other countermeasures against COVID-19 infection
- Evidence of increased transmissibility and severity of the virus

#### 2.1.3. Variants of High Consequence (VOHC)

Variants capable of increasing the virulence with corroborated proof on the decrease in the effect of treatments or vaccinations or evidence of reinfection in people who are already fully vaccinated. Currently, no such variant has been found.

Since late summer, the continued struggle with the Delta variant and emergence of highly transmissible Omicron variant have pushed the caseloads of different countries to the highest levels.  Figure 4 depicts the hotspots of the reported SARS-COVID-19 cases ranging from 10,000 to 10 million, with the size of the bubble determining the magnitude of the reported infected COVID-19 cases.

### 2.2. Testing for COVID-19 Infection

Due to the similarity of SARS-COVID-19 with normal flu and pneumonia, testing an individual for COVID-19 is a need to manage the disease effectively. Testing has played a vital role in the first wave of pandemic and continues to do so in the second wave throughout the world to detect whether an individual has contracted the virus or not. Testing an individual for COVID-19 can help identify a disease for many asymptomatic and presymptomatic carriers who drive the pandemic silently without developing any symptoms for a more extended period. There have been a lot of studies that have marked asymptomatic and presymptomatic individuals as significant carriers of the infection, contributing silently to more than 35% of the COVID-19 infections worldwide. The testing techniques for COVID-19 testing, as depicted in Figure 3, fall into two broader categories (Figure 5), viz., diagnostic tests and serology blood tests/antibody tests [20].

#### 2.2.1. Diagnostic Tests

These tests are responsible for diagnosing whether an individual is COVID-19 positive. Diagnostic tests directly diagnose the presence of virus in nasal or throat swabs; therefore, diagnostic tests are sometimes referred to as direct tests. Diagnostic tests for COVID-19 can be further subdivided into two categories [21].

*(1) Reverse Transcription Polymerase Chain Reaction (RT-PCR)*. RT-PCR (reverse transcription polymerase chain reaction) tests, also commonly known as molecular tests, are responsible for detecting the virus in the nasal or throat swab sample collected from a suspected individual. This test works by investigating the presence of COVID-19 RNA (ribonucleic acid) in the sample so collected. If found, this RNA (ribonucleic acid) is converted into DNA (deoxyribonucleic acid) using reverse transcriptase. The resulting DNA (deoxyribonucleic acid) strand is amplified several times to predict the presence of COVID-19 infection in suspected individuals accurately. These tests have specificity and accuracy of more than 75%; however, several studies suggest false negatives reported by RT-PCR (reverse transcription polymerase chain reaction) tests. This might be attributed to the mutations in COVID-19 strains [22].

*(2) Rapid Antigen Tests*. These tests are responsible for identifying COVID-19 antigens in the throat or nasal swabs collected from a suspected individual. These tests, however, have more chances of missing out on an active COVID-19 infection than RT-PCR (reverse transcription polymerase chain reaction) tests because of their low sensitivity. For example, suppose individual tests negative in the COVID-19 rapid antigen test report; confirmation on the same needs to be done using the RT-PCR (reverse transcription polymerase chain reaction) test. The test results for rapid tests are usually available within 1 to 2 hours of testing [23].

#### 2.2.2. Serology Blood Tests/Antibody Tests

These tests, unlike the diagnostic tests, can detect whether an individual was previously inflicted with COVID-19 infection or not. Antibody tests are responsible for detecting the presence of antibodies in the blood sample taken from a suspected individual. If the subject under study shows a positive antibody test report, it means that the individual has been affected by the virus sometime in the past. The presence of antibodies in the blood sample results from natural immunity (if the person is not vaccinated) or an immune response generated by the immune system to fight against the infection. These tests might also prove useful to investigate the effect of different types of vaccines developed for COVID-19. However, these tests fail to diagnose an active COVID-19 infection [24].

### 2.3. Vaccines for COVID-19 Infection

With the global race for vaccine intensifying, vaccination drive has kick-started for people over 18. In contrast, many in the 45+ age category are lining up to receive their second doses. The news of immunization has raised hopes for people vulnerable to the dangers of the pandemic for the current, deadlier second wave [25]. There are four different categories of vaccines (Table 2) available for combating the COVID-19 virus [26].

#### 2.3.1. Whole Virus Vaccines

These vaccines activate the immune system against the antigen through antibodies and T-cell production, thus playing a pivotal role in targeting it. When an individual gets exposed to the same virus somehow, the body's immune system gets primed, fighting off the infection. Sinovax is an example of the whole virus vaccine.

#### 2.3.2. Protein Subunit Vaccines

Novavax for COVID-19 falls in the category of protein subunit vaccines. These vaccines employ a different strategy of using spike proteins of the virus to produce immunity. Still, the small size of the viral fragment can be an issue as it can surpass our immune system unnoticed. Therefore, these vaccines involve the use of multiple vaccine shots in combination with a chemical adjuvant, thereby enhancing the capability of the vaccine to produce an immune response at a measurable rate.

#### 2.3.3. Viral Vector Vaccines

Sputnik-V, Covishield-Oxford-AstraZeneca vaccine, and Johnson and Johnson are proven to stimulate more robust immune responses by inserting genetic code for antigen by employing virus as a delivery system to deliver the code into the cells effectively.

#### 2.3.4. Nucleic Acid Vaccines

DNA (deoxyribose nucleic acid) and mRNA (messenger ribonucleic acid) vaccines fall into the nucleic acid vaccines category. The insertion of genetic code through attachment to molecule directly or by using a gene gun to produce antigens, thereby replacing the need of using virus directly as a delivery system, seems to be the baseline rule for the operation of these vaccines. Pfizer-BioNTech and Moderna are examples of mRNA (messenger ribonucleic acid) vaccines for COVID-19 with reported efficacy of 98%.

The COVID-19 pandemic remains a grave concern even after years of its upsurge. The consecutive waves of the pandemic continue to rage on in full force, ravaging different countries with a vengeance. The alarming rate of confirmed, infected, and death cases continue to see an upward trend, and if not controlled, the entire world will come to a halt sooner than expected, as is clear from rising numbers. The unprecedented and uncontrolled surge in cases in the second wave is attributed to the double variant mutant E484Q and L452R in the B.1.617 COVID-19 strain [27]. The Delta variant, first detected in India in December 2020, remains the most problematic version of the SARS COV-2 virus accounting for nearly all the COVID-19 infections globally, fueled by the unchecked spread of the novel COVID-19 infection in different parts of the world. There is an incredible degree of collaboration on the science side, with hundreds of hospitals worldwide gathering data in real-time to treat patients inflicted with COVID-19 infection on a priority basis. As far as the development of vaccines is considered, different countries of the world are working together to develop new vaccines for containing the COVID-19 spread.

However, despite such an unprecedented collaboration on the development and deployment of vaccines, COVID-19 pandemic is still far from over [28].

Several variants of COVID-19 have been reported. World Health Organization (WHO) classifies Delta as a variant of concern capable of increasing transmissibility, causing more severe disease, or reducing the effect of treatment and vaccines. Though capable of preventing or mitigating the severity of the illness and death, the current vaccines fail to block the infection completely. The virus can still replicate in the nose, even among the vaccinated people who can then transmit the disease further within a population. Henceforth, a new generation of vaccines is required to block the transmission of the infection. For the successive waves of COVID-19 hitting different countries, it has been concluded that outbreaks were easier to contain in places with well-functioning testing and tracing systems to quickly catch further episodes before they swell into more infection waves. The countries which succeeded in controlling the reproductive rates and infection rates of COVID-19 in the first wave performed better at mitigating the effects of consecutive waves [29]. Therefore, there is a need to build appropriate modeling strategies with prediction to help the government contain the successive waves of the COVID-19 pandemic with ease and success to ensure minimal loss of lives whilst keeping a check on the rate of transmission of the disease [30].

Globally, the vaccine doses administered (see Figure 2) for different countries remain scarce. However, several additional booster doses have been given to fully vaccinated individuals with the emergence of viral variants.

The following research demonstrates a systematic literature review (SLR) of the articles [31] published between December 2019 and June 2021. In addition, we incorporated a series of inclusion and exclusion criteria to produce infographic tables reviewing the state-of-art techniques to collate information employing COVID-19 prediction modeling. The findings of SLR will help the government and the healthcare practitioners to use the best prediction model governed by the highest prediction accuracy and other performance metrics to contain the successive waves of the COVID-19 pandemic in the future and prevent overwhelming the limited medical healthcare resources.

## 3. Methodology for Systematic Literature Review (SLR)

Systematic literature review (SLR) is an organized and systematic process for identifying, evaluating, and critically analyzing relevant research and collecting and analyzing data from studies that might be used in our study. The objective of SLR is to offer a comprehensive insight into current research on the formulated research questions. An SLR activity is governed by the development of a review protocol in the planning phase, which consists of five primary stages, viz., formulation of research questions, design of search strategy, and assessment of the literature for quality, procurement of data, and coalescence of data (Figures 6 and 7). The first stage consisted of identifying or formulating well-defined research questions within the scope of SLR. The keywords and terminologies were identified, and it was ensured that the research questions or the previous studies were not duplicated in the current SLR. In the second stage, we formulated a search strategy focusing on the studies relevant to the research questions developed in the first stage. This involved formation of a search string using the keywords identified in the first stage and the searching of the identified databases relevant to the topic of research. The third stage comprised of the selection of study describing the inclusion and exclusion criteria for conforming to whether the current research article(s) need to be included for the current SLR or not. The identified articles were subjected to a quality assessment procedure, which included the development of quality checklists to aid in the evaluation.

The fourth stage consisted of data extraction from the included studies governed by the inclusion and exclusion criteria decided upon in the third stage. A data extraction form refined through a pilot study was developed in this stage. Finally, the fifth stage involved data coalescence as per their addressal to the research questions identified in the first step [31].

### 3.1. Identified Research Questions

To elucidate and outline pragmatic evidence on mathematical modeling and machine learning models employed for COVID-19 spread, the current SLR will facilitate to answer the following set of formulated research questions:

IRQ1: Which machine learning techniques and compartmental models have been used for predicting the future course of COVID-19?

IRQ2: What is the overall accuracy of the prediction models so employed?

IRQ3: What are the critical disease-related parameters and most effective intervention strategies deployed for mitigating the spread of COVID-19 infection?

IRQ4: Are the vaccines developed so far effective against all the mutant COVID-19 strains?

IRQ5: Is the proliferation of COVID-19 an open issue to continue the research path?

### 3.2. Design of Search Methodology

The subsequent sections focus on the design of the search methodologies used for this study, including search keywords, literature repositories, and the search procedure.

#### 3.2.1. Blueprint of Search Strategy

The search strategy was formulated in the five consecutive steps listed below [31]:

- Deduction of essential keywords from the research questions
- Determination of alternate typos and synonyms for key phrases
- Lookup for relevant terms in related articles or literature
- Employing the Boolean OR operator to combine different typos and analogies
- Connecting the significant word using the Boolean AND

#### 3.2.2. Search String

2019-nCoV “ OR” COVID-19 “OR “SARS-CoV-2” OR “HCoV-2019” OR “hcov” OR “NCOVID-19” OR “severe acute respiratory syndrome coronavirus 2” OR “severe acute respiratory syndrome corona virus 2” OR “coronavirus disease 2019” OR ((“coronavirus” OR “corona virus”) AND (Wuhan OR China OR novel)) AND “Covid-19” AND “Mathematical Modelling” AND “Artificial intelligence” AND (techniques OR models) AND (Vaccines OR “Herd Immun∗” OR “Reproductive rate” OR “Asymptomatic” OR “Machine learn∗”) AND (“SIR Model∗ OR Quarantine OR Lockdown).

#### 3.2.3. Identified Databases and Search Engines

Six electronic databases, viz., PubMed, Springer Link, IEEE Explore, Web of Science and Google Scholar, Science Direct, and Web of Science, were used as the sources of information for collating articles related to the COVID-19 pandemic (Figure 8). An electronic catalog, bibliotheca Wiley (https://onlinelibrary.wiley.com) was used to gather relevant to our SLR. The search period was restricted from 1^st^ December 2019 till 15^th^ October 2021 as the first case of COVID-19 was reported in Wuhan, China, in early December 2019. While conducting this systematic review, Wiley contained 3,729, 226,555, and 345,446 research articles, nearing 575,730 articles on COVID-19. This bibliotheca provided filtering of the relevant articles based on the year of publication, researcher's name, category of research, type of publication, source title, and journal list.

The previously created search string was used to narrow the search in the specified databases. The preceding string was adjusted so that it could be included in various databases based on their syntax. All selected databases were searched using titles and keywords, full text, and abstracts; however, Google Scholar was searched using keywords and abstracts to minimize duplication of retrieved records.

#### 3.2.4. Search Process

To minimize the selection bias and the duplication of results, an effective and exhaustive well-organized search of all the relevant sources is a must for an SLR. Therefore, the initial search process (ISP) has been divided into two phases:

ISP1: This phase involves gathering the candidate set of articles collected by searching identified databases.

ISP2: This phase comprises the identification of relevant references from the candidate set of articles of phase 1 and the addition of the same to the articles of phase 1 if found apropos.

After applying these two initial search phases, Mendeley (http://www.mendeley.com) was employed to organize and manage the search results. The search process was further refined at each stage, subject to many scrutinizations as in Figure 8.

### 3.3. Article Selection

An enormous number of databases are available for extracting and gathering information related to the chosen domain of study. However, even after selecting specific databases for retrieval of articles, the duplication and irrelevancy in the search process conducted cannot be omitted. Therefore, there is a need further to refine the search study to the next level to minimize the selection of trivial articles. The study selection phase involves applying two steps, viz., inclusion and exclusion criteria and quality assessment check for finalizing relevant articles for study. The inclusion and exclusion criteria are used for the candidate set of articles gathered in the initial search phase 1 (ISP1) to facilitate the search results further.

Furthermore, the quality assessment criteria are established and practiced for these articles. This results in the selection of articles with a fair chance of answering the formulated research questions, which can then be employed to extract data. The secondary search is divided into the following two phases (Figure 8):

ASP1: this phase scrutinizes the candidate set of articles selected in the search process based on the inclusion and exclusion criteria. The articles possessing the capability to answer the formulated research questions are deemed relevant.

ASP2: this phase applies the quality assessment criteria on the set of relevant papers gathered in SSP1. Also, the set of relevant articles is searched for references relevant to the study. The resulting relevant articles found, if, any are added to the existing pool of articles.

#### 3.3.1. Inclusion and Exclusion Criteria

The following inclusion and exclusion criteria will furnish significant articles apt to choice of study for this SLR.

Inclusion criteria are as follows:

- Select those studies that employ either machine learning models, mathematical models, or both
- Include both the journal and conference versions of the articles
- The most recent and complete publications will be selected if there happen to be multiple duplicate publications of any article
- Include articles on COVID-19 from 1^st^ December 2019 till 30^th^ October 2021
- Select those articles that can answer at least one research question

Exclusion criteria are as follows:

- Exclude articles from books, workshops, symposiums, or articles under review
- Ostracize articles covering socioeconomic factors
- Articles that fail to answer even a single research question are excluded
- Rule out articles that are in the non-English language
- Exclude articles that do not prescribe any machine learning or mathematical modeling technique
- The initial search retrieved a total of 1178 candidate sets of articles. The investigation was further refined by applying inclusion and exclusion criteria which deemed 162 articles to be relevant. A secondary search was initialized for these articles to highlight the appropriate references and include relevant articles. It was concluded that secondary search led to the identification of 7 additional papers pertinent to the study taking the score of relevant papers to 169. Finally, a quality assessment checklist was applied to these articles, which fetched 50 articles as final for performing SLR (Figure 8). These articles were then used for the procurement of data

#### 3.3.2. Quality Evaluation of Selected Articles

Eight quality assessment questions were mapped out to evaluate the plausibility and relevance of the articles selected for study (Table 3). Three possible answers were calibrated for each question: yes, partly, and no. A scoring technique was employed on these quality questions where the answers could be scored as “Yes =1,” “Partly =0.5,” and “No = 0.” As a result, we obtained through the sum of all scores of responses to the quality assessment questions was deduced. The articles with a quality score greater than four were deemed relevant with an acceptable quality grade. This resulted in the exclusion of 114 articles and corroboration of only 50 articles of credible and valid grade (Table 4).

### 3.4. Threats to Validity

The gauging of threats to the review protocol's validity is critical to ensure that the final set of selected articles considered for review are of acceptable quality. Three primary challenges to the credibility of this review methodology have been reviewed, viz., article selection bias, publication bias, and probable information gathering inaccuracy.

The selection of publications for review involves the identification of key terms apropos to answer the formulated research questions. The next step consists of using subsequent strings or words for searching in the database engines identified for this SLR. However, it might so happen that titles, abstracts, or keywords of some relevant articles might not contain keywords in alignment with the aforementioned key terms.

In order to avert this bias in article selection, a manual search of COVID-19 articles in dimensions was conducted to ensure that the chances of missing out on papers relevant to this review are minimum. Also, the lookup of significant references in the selected papers and the application of inclusion and exclusion criteria in strict compliance with the identified research questions helped curb this threat to a reasonable extent. Finally, two reviewers were assigned for study selection, and the disagreements among them were resolved through consensus to stave off the study selection bias further. However, it is plausible that some of the relevant studies might be overlooked. We presume the numbers so reported to be relatively small for such cases.

Publication bias in the form of outcome reporting bias, gray-literature bias, and language bias is bound to coexist in our research. For example, outcome reporting bias dictates the publishing of positive results concerning probabilistic models in more numbers than negative results, leading to overestimating performance results. To alleviate the outcome reporting bias, some of the chosen articles report both positive and negative comparisons concerning applying the different probabilistic models employed for publication. In addition, the exclusion of gray literature (government reports, thesis reports, etc.) paves the way for the existence of publication bias ineluctably.

Finally, to suppress the risk of inaccurate extraction of information, a reevaluation scheme was enforced on the selected articles to identify true positives. This situation arises when the title of the chosen study dictates significance, but the contents are deemed insignificant to answer the formulated research questions. A quality assessment criterion was established through the formulation of quality assessment questions. All the authors rated the quality questions independently and reached consensus, resolving conflicts and achieving similarity in the context of rating.

### 3.5. Data Extraction and Synthesis

The application of the quality assessment criteria on the selected set of articles furnished 50 articles of considerable quality. These articles were subjected to data extraction procedure to fetch the following significant information, viz.,

1. Techniques employed for modeling COVID-19 data
2. Stipulated time for which the dataset was considered
3. Continent/country and region for which the prediction model was developed
4. Key epidemiological parameters, viz., cumulative case numbers, deaths and recovery rates, reproductive ratio (R0), case fatality ratio (CFR), and herd immunity for the assumed prediction interval
5. Asymptomatic or presymptomatic infections account for nearly 58% of the infections in the first wave of COVID-19
6. Type of intervention measures, viz., quarantine, hospitalization, testing, social distancing, facemasks, and their reported effectiveness on the control or mitigation of COVID-19
7. Effectiveness of developed vaccines against different variations of mutating COVID-19 strain
8. Number and type of performance metrics used to validate the proposed model(s)

In order to extract and gather information from the selected articles to answer the different research questions, two types of data synthesis techniques were employed, viz., narrative synthesis, reciprocal translation, and indirect translation. For addressing RQ1 to RQ3, narrative synthesis was employed, to display and disseminate the data on the identified research questions. In addition, different types of charts, viz., pie charts and bar graphs, were used to enhance the representation of the extracted data. For RQ4, reciprocal translation was used wherein different vaccines, viz., BNT162b2, ChAd0x1, and mRNA-1273, were tested for their effectiveness against B.1.1.7 and B.1.617.2 variant of COVID-19. The reciprocal translation is a technique used in data synthesis when synthesis can be accomplished by “transforming” each instance into each of the other cases when studies are on comparable items, and analysts are aiming to produce an additive summary. For example, for RQ4, Bernal et al. [77] evaluated and compared BNT162b2 and ChAd0x1 on B.1.1.7 and B.1.617.2 variants and confirmed a 94% effectiveness of BNT162b2 (2 doses) for B .1.1.7 variant and 80% effectiveness with B.1.617.2. Likewise, Pouwels et al. [80] considered the impact of BNT162b2, ChAd0x1, and mRNA-1273 on B.1.617.2 variant for U.K. and signified a 75%, 80%, and 95% effectiveness of the aforementioned vaccines for B.1.617.2 variant. This leads to the generalized result that “The vaccines BNT162b2, ChAd0x1 and mRNA-1273, are all effective against on B .1.1.7 and B.1.617.2 Covid-19 mutant variants with varying degrees of effectiveness.” For RQ5, indirect translation from RQ4 was used.

## 4. Results and Discussion

### 4.1. Characteristics of Selected Articles

*Modeling approaches*, *key epidemiological parameters*, and *intervention strategies* for COVID-19 are as follows: different modeling approaches were proposed, evaluated, and analyzed for articles under study (Figure 9). These models were classified into four categories: data-based mathematical models, machine learning models, ARIMA and regression, and hybrid models.

#### 4.1.1. Data-Driven Mathematical Models

Compartmental models assign a group of populations to different labeled compartments for modeling an infectious outbreak [39]. These models employ a mix of complicated integrodifferential mathematical equations, thereby aiding in the realization and plotting of various disease-related parameters, viz., infection rates, recovery rates, incubation period, latent period, and reproductive rate [40]. In addition, the impact of different intervention strategies, viz., quarantine, lockdown, and travel restrictions, can also be studied using these models by incorporating the appropriate compartment in the basic SIR model.

#### 4.1.2. Machine Learning Models

Different machine learning algorithms, viz., support vector machines (SVM), random forests (RF), gradient boosting trees (GBT), logistic regression, and neural networks might be employed to predict the chance of COVID-19 infection in a population (Figure 10). To effectively track COVID-19 patients in hospitals at early stages, as shown in Figure 5, X-ray images of patients are scanned with the help of efficient machine learning algorithms, and this has assisted in clinical decision making at the early stages of the pandemic throughout the world [41, 42]. The use of machine learning algorithms not only limits the burden on limited healthcare resources but also helps deliver better treatment outcomes [43, 44]. ML-based algorithms are also capable of discerning patients with mild and severe symptoms to expose them to different stages of treatment as per the seriousness of the disease. For example, in the current COVID-19 scenario, the deployment of robots in hospitals to monitor patients' symptoms and deliver drugs to them thereby minimizes the exposure risk of healthcare practitioners to the virus [45].

#### 4.1.3. Autoregressive Integrated Moving Average (ARIMA) and Regression

This category combines two statistical models, viz., regression and Autoregressive Integrated Moving Average (ARIMA) into one for forecasting future infections. The resulting model enticed as regression with ARIMA corrections enhances the performance and reliability of predictions.

#### 4.1.4. Hybrid Models

The synergy of data-driven mathematical modeling and machine learning algorithms might be a boon for healthcare practitioners to develop optimal policies to control or mitigate the spread of COVID-19 in various settings [59]. The mathematical formulae devised using statistical modeling can help predict the future course of infections which can aid in optimal policymaking. Different machine learning algorithms, viz., support vector machines (SVM), random forests (RF), gradient boosting trees (GBT), and logistic regression can work efficiently in tandem and close proximity with explicit differential equations devised through modeling that might help in future forecasting of the pandemic as shown in Figures 2 and 6, based on historical patterns of data in different settings [60, 61]. Incorporating various disease-related parameters and variables into statistical models might provide insights into the dynamics of disease transmission, and this might prove helpful in future forecasting of the disease. The models so developed through the integration of mathematics and AI technologies will help investigate the effects of various interventions like quarantine, testing, drugs, vaccination, and their relative impacts on flattening the curve.

Furthermore, the models mentioned above identified for prediction covered four aspects of study, viz., gaining insights into the transmission dynamics with or without predicting the course of COVID-19 infection in advance (infection rates, recovery, and death rates), metrics employed by prediction models for assessing performance, assessment of various disease-related parameters of COVID-19, the efficacy of reported vaccines on mutating COVID-19 strains, and gauging the impact of various intervention measures on the spread of COVID-19.

### 4.2. Which Machine Learning Techniques and Compartmental Models Have Been Used for Predicting the Future Course of COVID-19?

From the selected studies, 64% of the studies include mathematical models for modeling infections. Over 2.48% of the articles employed a single machine learning algorithms for study, whereas 26% employed multiple machine learning algorithms, viz., support vector machine (11%), random forest (6%), decision trees (4%), gradient boosting algorithm (3%), AdaBoost (1%), and XGBoost (1%) (Figure 10). Nearly 40% of the articles studied and calibrated the basic SIR model, with around 35% of the models predicting the trend of this infectious spread. Around 30% of the selected studies modeled the effect of various intervention measures, viz., lockdown (8%), quarantine (16%), travel restrictions (3%), asymptomatic cases (3%), and on the infection rates (Table 5).

The selected studies constituted only 5% of hybrid models employing compartmental and machine learning algorithms. It is concluded that around 43% of the chosen studies predicted the trend of COVID-19 spread, whereas 38% of the articles focused on the study of various parameters, viz., reproductive rate (26%), case fatality ratio (6%), herd immunity (4%) concerning epidemiology, and their effect on curbing the infection rates or flattening of COVID-19 infection curve. Also, ARIMA and regression accounted for nearly 3% of the articles under study.  Figure 11 portrays the forecasting dynamics employed by the different articles under study.

### 4.3. What Is the Overall Accuracy of the Prediction Models Employed?

The articles selected for study employed either compartmental models or machine learning models or a combination of both to project the infection rates. For studies using mathematical modeling, viz., SIR, SIER, and SIRD models, the prediction accuracy is quite difficult to anticipate in advance. These models consider several assumptions while modeling, which may or may not go well with different settings. These assumptions are nothing but idealization and approximation of what is happening in reality. Therefore, it is vague to expect valuable predictions from such models, which are incapable of mirroring different facets of reality. For example, Lourenço et al. [48] employed a SIR (Susceptible, Infected, Recovered) model to study the severity of the spread of COVID-19 in the U.K. and Italy. The study predicts the infliction of 60% of the U.K. population with the virus by 19 March 2020 at R0 = 2.25. The SIR model dictates that the number of susceptibles S(0) should be marginally less than the ratio *a*/*b* to prevent an epidemic, where *a* is the recovery rate and *b* is the transmission rate. This implies that even before the arrival of mutant strains, a certain fraction of the population should be vaccinated to reduce the initial number of individuals susceptible to infection, thereby maintaining *S* (0) < *a*/*b*. However, this underestimates herd immunity which dictates that herd immunity can only be achieved if the pandemic spreads in more than 95% of the population. Also, Gupta [43] employed a SIER model to predict the future trend of COVID-19 in India for three weeks. However, the predictions made cannot be expected to be 100% accurate because of deviations, viz., underreporting of COVID-19 data, assumptions withheld while formulating the model.

Similarly, Kyrychko et al. [47] suggested a variation of the SIER (Susceptible, Infected, Exposed, Recovered) model to model the effect of COVID-19 infection on recovery and death rate in Ukraine. The study suggested an increase in both infection and death rates with time without appropriate mitigation strategies in individuals with the age group 60-70. However, later, it was found out that young people within the age group 25-35 were the most affected. Therefore, it is difficult to anticipate the reliability of such predictions. Furthermore, the mathematical models of [51] assume a homogenously mixing population, which is quite vague as it is implausible that all individuals have an equal probability of getting in contact with other individuals. Also, the model of [55], which has been validated for a large population, might fit well for cities. Still, the deduction of results through different equations will lead to unrealistic results for villages.

Moreover, the results of [59] assume an exponential distribution of infection and overlook the period from the onset of symptoms to recovery or death, which is quite unrealistic. For studies employing more than one model for prediction, the fitted parameters and results deduced might be considered valid and robust, for example. Still, the notion of prediction for referring parameters dictated by the model should be restricted for studies relying on only one model.  Table 6 depicts the Quality Evaluation Metrics employed by the articles selected for SLR of COVID-19.

Nonetheless, the benefit that these mathematical models offer in terms of early prediction of infection, death, and recovery rates and the development of policies as far as control of pandemic is concerned cannot be overlooked. Several mathematical models employed the technique of multiple factor optimization to account for the bias in calculations caused due to underreporting of data. For example, Anastassopoulou et al. [52] employed the SIRD (Susceptible, Infectious, Recovered, Dead) model to study the effect of various parameters, viz., CFR (case fatality ratio), R0 (reproductive ratio) related to COVID-19 epidemiology on the infection, death, and recovery rates for Hubei, China. The projected average value of R0 is determined to be 2.6, premised on SIRD simulations. The simulations have been repeated by considering the number of infected cases multiplied by a factor of 20 and the number of recovered cases multiplied by 40 to account for the bias in calculations caused due to underreporting of asymptomatic or presymptomatic patients. Around 38% of the compartmental models employed for studying the dynamics of COVID-19 include stability and sensitivity analysis of various parameters to account for the division and allocation of different sources of uncertainty in inputs to the uncertainties of the output to justify the reliability of results. These models are quite helpful while incorporating the effect of various intervention strategies, viz., lockdown, quarantine, and the role of international travel, on the curve of epidemic. To gauge the accuracy of mathematical models, while some parameters are assumed, others are deduced by fitting the model with datasets.

With a view to gauge the capability of prediction models for the spread of COVID-19 employing machine learning, modeling has to be guided by performance metrics. These evaluation metrics enable the quantification of performance dictated by machine learning models. Different algorithms are elucidated, and hyperparameters are tuned with the involvement of a distinct set of decided-upon features. Accuracy, precision, ROC/AUC, sensitivity, specificity, F1 score, recall, and Brier score are some of the performance metrics for evaluating the developed predictive model. More than 80% of the ML models employed for COVID-19 spread use specificity, sensitivity, accuracy, precision, and recall to evaluate performance. Hassanein et al. [38] suggested the use of SVM (support vector machine) to diagnose whether an individual is inflicted with COVID-19 or not. The reported accuracy, specificity, and sensitivity of 97.5, 99.7, and 95.8 have been reported. Likewise, De Moraes [39] studied SVM, RF, GBT, and logistic regression for COVID-19 spread. Out of all these algorithms, SVM and random forest reported similar AUC, sensitivity, and specificity of 0.851, 0.677, and 0.850.

### 4.4. What Are the Essential Disease-Related Parameters and Most Effective Intervention Strategies Deployed for Mitigating the Spread of COVID-19 Infection?

The probabilistic models employed for understanding the dynamics of COVID-19 spread have been used to deduce several disease-related parameters, viz., case fatality ratio (CFR), reproductive rate (R0), transmission rates, infection rates, recovery rates, asymptomatic infection rate, and herd immunity (Figure 12). In addition, several control measures and their effect on the infection rates have been studied (Figure 13). Around 45% of the developed models incorporated the estimation, assumption, and effect of varying R0 of COVID-19 to gain insights into the transmission dynamics of COVID-19, whereas only 3% of the selected articles focused on the deduction of CFR, an important parameter for understanding the severity of the disease. McGoogan and Wu [32] estimated the CFR in China to be equal to 2.4% on 12^th^ February 2020. Also, Wu. et al. [34] employed a SIER model for understanding the trend of infectious spread of COVID-19 for major cities of China and deduced R0 to be roughly equal to 2.7 using Monte Carlo simulations. Read et al. [35] studied the early estimation of various parameters and predicted R0 = 3.1 assuming Poisson's distribution for the infectious cases in Wuhan, China.  Table 7 lists multiple disease-related parameters and intervention measures considered by the articles under study. Estimating infection and death rates for a predefined interval is an important exercise to ensure well-preparedness in advance for mitigating COVID-19 infection. Around 39% of the selected studies model the infection and death rates of COVID-19.

Anastassopoulou et al. [52] considered a SIRD model for simulating the total number of infections and predicted the number of infections to cross 2 lakhs by February. Also, the death toll is expected to cross 2,800 by the end of February 2020. Around 3% of the studies modeled the effect of asymptomatic individuals on the growth curve of the epidemic. The time-varying SIR model of Peng et al. [68] confirmed a 20% contribution of asymptomatic infections to the total infections. Also, Tomochi and Kono [49] included a compartment I in the basic SIR model and reported asymptomatic infections to account for 15% of the COVID-19 infections.

Around 45% of the models considered for the projection of infection rates studied the effect of quarantine on the infected cases. Zhong et al. [37] predicted a reduction in peak infectives by 40-50% through the deployment of quarantine regime at 20% in China. The lockdown and social distancing regime is modeled by around 25% and 13% of the selected articles. Khan et al. [50] concluded that a reduction in contact rate by 11% or doubling the rate of lockdown will effectively eradicate the infections in the U.S. within a year. Grimm et al. [59] employed a variation of the SEIR model to study the effect of social distancing and the use of tracing applications on daily reported infections and deaths.

The study concluded a 60% reduction in infections through the implementation of social distancing alone. Mandal et al. [54] employed variation of SIR (Susceptible, Infectious, Recovered) model called the SEQIR model to predict the effect of quarantine on the reproductive ratio, R0 a vital indicator in epidemiology to understand the trend of COVID-19 transmission. The results deduce that increasing the duration of quarantine or isolation rate will slow down the spread of disease transmission by cutting R0 below 1. Feng et al. [60] employed the SEIR (Susceptible, Infected, Exposed, Recovered) model to study the trend of COVID-19 spread in Wuhan from 23^rd^ January 2020 to 6^th^ March 2020. The study predicts the total number of positive cases to cross the 40,000 mark in the next seven days from the included time interval by fitting the various parameters of the SEIR model as per the reported data. The study also focuses on the effect of quarantine on the mitigation of COVID-19 spread. It concludes that there will be an increase in the number of cumulative cases for Beijing and Henan in the absence of quarantine by 1.8 times within 3.5 weeks.

### 4.5. Are the Vaccines Developed So Far Effective against All the Mutant COVID-19 Strains?

An overall drop in cases seen at the end of December 2020 led to the relaxation in lockdown restrictions; however, soon, new variants of COVID-19 started showing in different countries. Specific mutations of the COVID-19 virus were reported that were capable of binding human receptors better and at a fast pace. COVID-19 viruses are covered in spike proteins used for binding and infecting human cells. As a result, multiple variants started emerging in different places around the globe, viz., alpha (B.1.1.7), beta (B.1.351), gamma (P.1), and delta (B.1.617.2). The Delta strain was considered the worst of all the COVID-19 mutant strains and was referred to as “double mutant” because of two different mutations, L452R and E484Q (E484K). E484Q and E484K can induce reinfection in people already infected with COVID-19, i.e., these two mutations have evolved to dodge the natural immune response.

The selected studies conclude that B.1.617.2 has the potential to cause breakthrough infection even in the presence of vaccine-induced or natural immunity. As a result, different types of vaccines and their efficacy against alpha and delta variants have been studied. Bernal et al. [77] studied the effect of Pfizer-BioNTech (BNT162b2) and Oxford-AstraZeneca (ChAd0x1) on B .1.1.7 variant (Figure 14) in U.K. The study concluded a 73% effectiveness with ChAd0x1 after 30 days, whereas the same reduces to 61% with BNT162b2 for the same baseline interval. Tang et al. [78] assessed the effectiveness of Moderna (mRNA-1273) and BNT162b2 on the B.1.617.2 variant and found mRNA-1273 to be 100% effective (14 days after the second dose). In contrast, Pfizer was only 90% effective against the B.1.617.2 COVID-19 variant.

Bernal et al. [79] evaluated and compared BNT162b2 and ChAd0x1 on B .1.1.7 and B.1.617.2 variants and confirmed a 94% effectiveness of BNT162b2 (2 doses) for B.1.1.7 variant, whereas the impact significantly reduced to 10% for those inflicted with B.1.617.2 (Figure 15). This concludes that while the vaccines show a decrease in their efficacy against the B .1.1.7 and B.1.617.2 variants and chances of getting reinfections with both the variants; however, protection of 80-90% is still expected with vaccine-induced antibodies.

Pouwels [80] considered the impact of BNT162b2, ChAd0x1, and mRNA-1273 on B.1.617.2 variant for U.K. and signified a 13%, 14%, and 16% decrease, respectively, for the aforementioned vaccines for B.1.617.2 variant. Thus, there is a decrease in the severity of disease in terms of symptoms developed with both B.1.1.7 and B.1.617.2 variants; however, B.1.617.2 (see box plot of Figure 16) is more capable of neutralizing vaccine-induced antibodies than the B.1.1.7 variant.

### 4.6. Is the Proliferation of COVID-19 an Open Issue to Continue the Research Path?

The COVID-19 virus is mutating at a fast pace. The Delta variant is classified by the World Health Organization (WHO) as a variety of concern capable of increasing transmissibility, producing more severe illness, or limiting the effectiveness of therapy and vaccinations [77]. While capable of avoiding or lessening the severity of the disease and mortality, the present vaccinations do not block the infection completely.

The new COVID-19 variant Omicron (B.1.1.529) has been identified in South Africa, and it has become a sauce of concern for many countries in terms of its virulence and transmissibility. This variant carries 50 mutations (32 on spike protein) which could further drive the consecutive waves of the COVID-19 while Delta had two mutations only, and the same is confirmed through genome sequencing. India has reported 100 cases of Omicron variant just after 15-20 days of the first identified case in South Africa, which is quite alarming [78]. This variant has sent menacing shock waves across countries. Unvaccinated individuals remain at high risk of intense symptoms. Also, this mutant evades vaccine immunity; hence, additional booster shots are given to enhance the presence of antibodies [79]. Multiple cases of the Omicron variant (B.1.1529) have been reported in Botswana, Hong Kong, and South Africa. There is a sudden surge in the reported case numbers by 12%. The Delta and Omicron variants are driving the fastest surge of new COVID-19 cases in Africa, with about 196,000 new cases reported per week. The number of infections has increased tenfold since the start of October 2021.

The Omicron variant is spreading faster with a doubling time between 1.5 and 3 days (Figure 17) in countries with documented community transmission. Omicron has a substantial growth advantage over delta [15]. The number of infections has increased tenfold since October 2021 (Figure 18). There is a sudden surge in cases and probably an increase in hospitalizations and deaths, thereby draining the hospital capacity (Figure 19). Booster campaigns and new social restrictions might help in keeping the infections at bay. The quarantine regime is again followed for individuals traveling from the affected countries where the individuals inflicted with this mutant strain have been found, and WHO suggests the widespread use of boosters for protection against this variant. As such, COVID-19 is far from over.

The shared data is playing a pivotal role in the global efforts to combat the spread of COVID-19. Therefore, there needs to be a collaboration on public and private platforms to review the global data for testing potential, treatment vaccines, and therapeutics [79], and the more the research concerning the different facets of COVID-19 spread, the more the expertise gained at developing optimal solutions to roadblock the progression of COVID-19. Henceforth, this justifies the need for continuous research focused on mitigating the effects of virulent replicating strains of COVID-19 [81].

## 5. Limitations of the Conducted SLR

The different ML models employed by the articles considered for this SLR have included different performance metrics to evaluate the accuracy of the prediction models. Besides this, several other factors contributing to the accuracy, viz., generality, decipherability, and accountability, have not been considered by this review. Due to the difference in experimental designs, the accuracy of reported results is difficult to anticipate, subject to the conditions taken into account while generalizing models. No comparison between ML and mathematical models has been contemplated. This inconsistency might be attributed to the limited number of articles considered for this study. Also, the compartmental models reviewed employ many assumptions while modeling the COVID-19 pandemic. However, these assumptions change with the emergence and availability of new data. With this, projections are subject to change; hence, one model might be plausible under certain conditions but might be deemed unfit in other scenarios. No metric has been evaluated/reported to gauge this inconsistency. The reported mathematical predictions, viz., infection numbers vary significantly with the changing nature of mutating COVID-19 viral strain, which questions the understandability, application, and reliability of these models in different scenarios. Some accentuating limitations of this SLR are as follows:

- GIGO (Garbage In, Garbage Out) was overestimated while performing this SLR
- Heterogeneity concerning statistical assessment was outperformed in the current SLR
- Meta-analysis methods were underestimated in the studies selected for conducting this SLR
- Nonstandardization of assessment methods in the studied articles could not be wholly avoided
- Generalization of results from an SLR to contexts not studied would report issues
- Publication and language bias could not be completely eliminated
- The reported results were sensitive to the size of the studies selected for this SLR

## 6. Conclusion

Predictive modeling is a must to contain the devastating delta strain of the virus at this lethal stage of COVID-19. The reported results from SLR encompass and summarize diverse models and techniques used for analyzing the dynamics of the spread of COVID-19. Around (35%) of the selected studies enlisted dynamics reporting COVID-19 case numbers, (30%) modeled the effect of intervention measures, and (20%) estimated the different disease-related parameters concerning COVID-19. Only (10%) and (5%) of the studies focused on testing strategies and vaccine effectiveness, respectively, for COVID-19. The current SLR shows a positive effect of BNT162b2, ChAd0x1, and mRNA-1273 on B.1.1.7 and B.1.617.2 viral variants and suggests administering additional booster doses for immunosuppressant individuals or normal individuals to make up for the deficit of waning antibodies given current continuously evolving new variants of COVID-19. Most of the models used 95% CI for predicting cumulative cases over a predefined interval. The findings of SLR suggest that predictions made by different models are essential to understand the course of the COVID-19 pandemic, subject to QEM used by each. The results from performance metrics used by each show that random forest (RF) and support vector machine (SVM) performed better for predicting COVID-19 case numbers followed by decision tree (DT), linear regression, and gradient boosting algorithm (GBA).

Moreover, this systematic review suggests using the SIR model to incorporate various disease parameters. This would help in gauging the impact of different interventions for controlling the pandemic and modeling the vaccination, which seems to be the most important for this global emergency. However, given a scenario, it is pretty tricky to anticipate which model will perform the best because of the continuous change in the dynamics of the COVID-19 virus and the dataset chosen for study. The machine learning algorithms might be integrated with deep learning algorithms to project COVID-19 infection cases in advance, and mathematical modeling might be used to study the effect of control measures on the infection rates.

## Figures and Tables

**Figure 1:** Dynamics of transmission for the spread of SARS-Covid-19.

**Figure 2:** Graph depicting vaccination rates by region for SARS-COVID-19 [17].

**Figure 3:** SARS-COVID-19 cases per capita in different parts of the world from 28 February 2020 to 30 October 2021 [17].

**Figure 4:** Map depicting the known locations of cumulative reported SARS-COVID-19 cases [17].

**Figure 5:** Testing techniques for detection of SARS-COVID-19 [8].

**Figure 6:** Framework depicting different phases employed for current SLR on SARS-COVID-19 [31].

**Figure 7:** Flowchart depicting PRISMA-based stepwise methodology for the development of review protocol for current SLR [31].

**Figure 8:** Flowchart depicting identified databases and evaluation criteria for final selection of articles for current SLR on SARS-COVID-19 [31].

**Figure 9:** Chart illustrating percentage-wise model-type used for SARS-COVID-19.

**Figure 10:** Graph depicting the type of machine-learning techniques used for SARS-COVID-19.

**Figure 11:** Graph portraying dynamics of predictions for SARS-COVID-19.

**Figure 12:** Percentage-wise disease-related parameters reported by current SLR.

**Figure 13:** Control measures employed by the articles under study for SARS-COVID-19.

**Figure 14:** Reported vaccine effectiveness percentage against B.1.1.7 SARS-COVID-19 variant strain.

**Figure 15:** Reported vaccine effectiveness percentage against B.1.617.2 SARS-COVID-19 variant strain.

**Figure 16:** Plots showing reported efficacy of different vaccines for B.1.1.7 and B.1.617.2 COVID-19 mutant strains.

**Figure 17:** Different SARS-COVID-19 variants with their doubling time [15].

**Figure 18:** Graph depicting reported case numbers of SARS-COVID-19 for India variants from 28 February 2020 to 30 October 2021.

**Figure 19:** Trajectory for deaths due to the evolution of SARS-COVID-19 viral variants from 28 February 2020 to 13 December 2021.

**Table 1:** Description of SARS-COVID-19 mutant strains [7].

Variants of interest			
S. no.	WHO label	Lineage	First documented sample
1	Epsilon	B.1.427/B.1.429	U.S.A., March 2020
2	Zeta	P.2	Brazil, April2020
3	Eta	B.1.525	Multiple, Dec 2020
4	Theta	P.3	Philippines, January 2021
5	Iota	B.1.526	U.S.A., Nov 2020
6	Kappa	B.1.617.1	India, October 2020
7	Lambda	C.37	Peru, August 2020
Variants of concern			
1	Alpha	B.1.1.7	U.K., September 2020
2	Beta	B.1.351	South Africa, May 2020
3	Gamma	P.1	Brazil, November 2020
4	Delta	B.1.617.2	India, October 2002
5	Omicron	B.1.1.529	South Africa, November 2021
Variants of high consequence (none identified)			

**Table 2:** Categories of vaccines for SARS-COVID-19 [9].

Vaccine category	Type/company	No. of doses	Other vaccines employing this technology	Storage
RNA	Pfizer-BioNTech Moderna	2	No other licensed vaccines	Pfizer-BioNTech: -70°C and 2-8°C for up to 5 days Moderna: -20°C for 6 months And 2-8°C for 30 days
Viral vector	Oxford-AstraZeneca CanSino Biologics Gamaleya Research Institute Johnson and Johnson	1-2	Ebola	2-8°C
Whole virus	Sinovac (inactivated) Bharat Biotech (inactivated)	2	Whooping cough (inactivated) Rabies (inactivated) Hepatitis A (inactivated)	2-8°C
	Sinopham (inactivated) Medicago Inc. (virus-like-particle)		HIPV/cervical cancer (virus-like-particle)	
Protein subunit	Novavax Chinese Academy of Sciences	2	Hepatitis B	2-8°C

**Table 3:** Quality evaluation questions for assessing the quality of selected articles.

Quality evaluation ID	Quality evaluation questions
QE1	Is there a clear articulation of the objectives of the undertaken research?
QE2	Are the predicted models justifiable and deliberate under a given context or setting?
QE3	Are the findings deliberated by the prediction models validated?
QE4	Are sufficient datasets employed for experimental setup?
QE5	Are the predicted models compared with others to ensure efficiency?
QE6	Does the study narrate its limitations?
QE7	Do the prediction models motivate academia to continue the chosen research path?
QE8	Is the accuracy of the predicted model(s) reported?

**Table 4:** Quality assessment scores for selected articles.

Article Id	Author	QE1	QE2	QE3	QE4	QE5	QE6	QE7	QE8	Total score
A1	Wu and McGoogan et al. [32]	1	0.5	0.5	1	0	1	1	0	5
A2	Bottcher et al. [33]	1	0.5	0.5	0	1	1	1	0.5	5.5
A3	Wu et al. [34]	1	0.5	1	0	0	1	1	0.5	5
A4	Read et al. [35]	1	0.5	1	0	0	1	1	0.5	5
A5	Hong et al. [36]	1	1	0.5	0	1	1	1	0.5	6
A6	Zhong et al. [37]	1	1	1	0	0	0	1	0.5	4.5
A7	Hassanein et al. [38]	1	0.5	1	0	0	1	0.5	1	5
A8	De Moraes et al. [39]	1	1	0.5	0	1	1	0.5	1	6
A9	Zoabi et al. [40]	1	1	0.5	0	1	1	0.5	1	6
A10	Farooq and Bazaz [41]	0.5	1	1	1	0.5	1	1	0	6
A11	Dos Santos Santana et al. [42]	1	1	1	0	1	1	1	1	7
A12	Gupta [43]	1	1	1	0	0	1	0.5	0	4.5
A13	Anderez et al. [44]	1	1	1	1	0	1	0.5	1	6.5
A14	Goodman-Meza et al. [45]	1	1	1	0	1	0	1	1	6
A15	Ndaïrou et al. [46]	1	1	1	1	0	1	0.5	0.5	6
A16	Kyrychko et al. [47]	1	1	1	1	0	1	0.5	1	6.5
A17	Lourenço et al. [48]	1	1	1	1	1	0	0.5	1	6.5
A18	Tomochi and Kono [49]	1	1	1	0	0	1	0.5	1	5.5
A19	Khan et al. [50]	0.5	1	1	1	0	1	1	1	6.5
A20	Hassan et al. [51]	1	1	1	0	0	0	1	1	5
A21	Anastassopoulou et.al [52]	1	1	1	1	0	0.5	1	1	6.5
A22	Saxena et al. [53]	1	1	1	1	0	0.5	1	1	6.5
A23	Mandal et al. [54]	1	1	1	1	0	1	0.5	1	6.5
A24	Saikia et al. [55]	1	1	1	1	0	1	1	1	7
A25	Hassen et al. [56]	1	1	1	1	0	0	1	1	6
A26	Nguemdjoid et al. [57]	1	1	1	0	0	0	1	1	5
A27	Munoz-Fernandez et al. [58]	1	1	1	1	0	1	1	1	7
A28	Grimm et al. [59]	1	1	1	0	1	1	1	1	7
A29	Fengid et al. [60]	0.5	1	1	1	0	1	1	1	6.5
A30	Sharpio et al. [61]	1	1	1	1	1	0	1	1	7
A31	Malavika et al. [62]	0.5	1	1	1	0	1	1	1	6.5
A32	Rahimi et al. [63]	1	1	1	1	1	1	0.5	1	7.5
A33	Gecili et al. [64]	0.5	1	1	1	1	0	1	1	6.5
A34	Alshomrani et al. [65]	1	1	1	1	1	0	0.5	1	6.5
A35	Chen et al. [66]	1	1	1	0	1	0	1	1	6
A36	Ala'raj et al. [67]	1	1	1	1	1	1	0.5	1	7.5
A37	Peng et al. [68]	1	1	1	1	0	0	1	1	6
A38	Shin [69]	1	1	1	0	1	0	1	1	6
A39	Li et al. [70]	1	1	1	0	1	0	1	1	6
A40	De La Sen et al. [71]	1	1	1	0	1	0	1	1	6
A41	Abbasi et al. [72]	1	1	1	1	0	0	1	1	6
A42	Khanday et al. [73]	1	1	1	1	0	0	0.5	1	5.5
A43	Mojjada et al. [74]	1	1	1	1	0	1	1	1	7
A44	Sen and Sen [75]	1	1	1	1	1	0	0.5	1	6.5
A45	Goo et al. [76]	1	1	1	0	1	0	0.5	1	5.5
A46	Lopez et al. [77]	0.5	0.5	1	1	0.5	1	1	1	6.5
A47	Tang et al. [78]	0.5	0.5	1	1	0.5	1	1	1	6.5
A48	Lopez et al. [79]	0.5	1	1	1	1	1	1	1	7.5
A49	Pouwels et al. [80]	0.5	1	1	1	0.5	1	1	1	7
A50	Mlochova et al. [81]	1	1	1	0	0.5	1	1	1	6.5

**Table 5:** Types of models employed for modelling SARS-COVID-19.

Author/reference	Major contribution	Type of model employed
Wu and McGoogan et al. [32]	Estimation of case fatality ratio (CFR) to assess the severity of COVID-19 for China.	Basic SIR model
Bottcher et al. [33]	Evaluation of factors influencing the population-based CFR's and individual-based CFR's at a constant recovery and death rate for China.	SIR model
Wu et al. [34]	Deduction of reproductive ratio, R0, to be roughly equal to 2.7 for Wuhan, China.	SIER model
Read et al. [35]	Early estimation of various parameters concerning epidemiology and predicts the value of the reproductive ratio, R0, to be 3.1 for China.	SIR model
Hong et al. [36]	Evaluating the value of R0 to enhance the effectiveness of various policies for early control of the pandemic for China.	SIR model
Zhong et al. [37]	Modeling the infection and removal rates of COVID-19 and prediction of the cumulative COVID-19 cases for China	SIR model
Hassanein et al. [38]	Detection of the presence of COVID-19 infection in the lungs at early stages.	SVM
De Moraes et al. [39]	Employing machine learning algorithms to prioritize the infected cases for receiving the RT-PCR (reverse transcription polymerase chain reaction) tests in case of limited testing resources.	Machine learning models: SVM, RF, GBT, and LR models
Zoabi et al. [40]	Prioritizing the infected cases for receiving the RT-PCR (reverse transcription polymerase chain reaction) in case of limited testing resources.	DT
Farooq et al. [41]	Understanding the trend of infectious spread for the worst-hit states of India.	SIR model
Dos Santos Santana et al. [42]	Prioritization of the infected cases for receiving the RT-PCR (reverse transcription polymerase chain reaction) tests in case of limited testing resources.	Machine learning models: SVM, RF, GBT, LR, and DT models
Gupta et al. [43]	Computation of reproductive ratio, R0, to predict the future trend of COVID-19 for three weeks' time.	SIER
Anderez et al. [44]	Modeling the mortality rate for people who are already vulnerable to infection due to their advanced age or existing combordities before getting exposed to the virus.	SIER
Goodman-Meza et al. [45]	Various features and different clinical diagnoses like complete blood counts (CBC's) and various inflammatory markers are studied to diagnose a person as being COVID-19 positive or negative.	Machine learning and ensemble models: SVM, LR, RF, AdaBosst, and XGBoost
Ndaïrou et al. [46]	Graphing the number of confirmed, recovered, and fatality cases using a dataset within a stipulated time period.	SIR model
Kyrychko et al. [47]	Exploration of the impact of lockdown strategies on infection and death rates.	SIER
Lourenço et al. [48]	Study the severity spread of COVID-19 via modeling of infections.	SIR model
Tomochi and Kono [49]	Modeling different parameters associated with COVID-19, viz., incubation period, reproductive number, effective reproductive number, the peak of infection, and herd immunity threshold.	SIIR model: incorporation of I compartment for modeling asymptomatic infections
Khan et al. [50]	Impact of lockdown strategies on infection and death rates.	SIER
Hassan et al. [51]	The study explores the impact of lockdown strategies on infection, recovery, and death rates.	SIRD model
Anastassopoulou et al. [52]	Modeling the effect of various parameters, viz., CFR (case fatality ratio), R0 (reproductive ratio) related to COVID-19 epidemiology on the infection, death, and recovery rates.	SIRD
Saxena et al. [53]	Study various parameters related to COVID-19 transmission, viz., contact rate, reproductive rate (R0), and range of COVID-19 spread.	SIER
Mandal et al. [54]	Prediction of the infection rates for three regions of India.	SIER
Saikia et al. [55]	Study the effect of asymptomatic infections on the transmission rate of the COVID-19.	SIER
Hassen et al. [56]	Modeling the different epidemiological parameters, viz., transmission rate and reproductive rate (R0) for COVID-19.	SIR
Nguemdjoid et al. [57]	Study the effect of various intervention measures on the pandemic's reproductive rate (R0) to flatten the curve of COVID-19.	SIR
Munoz-Fernandez et al. [58]	Study of the daily infections, transmission rates, and deaths due to COVID-19.	SIR
Grimm et al. [59]	Modeling the effect of various intervention measures on the mitigation of COVID-19 spread.	SEIR
Fengid et al. [60]	Prediction of infection and mortality rates.	SEIR
Sharpio et al. [61]	Estimation of the infection rates and reproductive rates (R0) of epidemic.	SIR model
Malavika et al. [62]	Prediction of the maximum number of active cases and study the effect of three-week lockdown and other intervention measures on the curve of COVID-19.	Logistic growth curve model and time interrupted regression model
Rahimi et al. [63]	Prediction of infection rates, reproductive rates, total confirmed and death cases.	Hybrid: SEIR and SVM
Gecili et al. [64]	Modeling the number of confirmed positive, recovery, and death cases for COVID-19.	Holt model, ARIMA, TBATS, cubic smoothing spline model
Alshomrani et al. [65]	Estimating various epidemiological parameters, viz., reproductive rate, transmission rate, and recovery rate by fitting the parameters.	SIR model
Chen et al. [66]	Study the effect of asymptomatic individuals on the spread of COVID-19.	SEIR
Ala'raj et al. [67]	Study the cumulative number of infectives, recovery, and death cases due to COVID-19.	SEIR with ARIMA corrections
Peng et al. [68]	Study the unreported infection rate (UFR), infection fatality rate (IFR), and transmission rate (TR) for COVID-19 cases.	SIR
Shin [69]	Modeling through multistage transitions to understand the dynamics of three successive waves of COVID-19 transmission.	SEIR
Li et al. [70]	Modeling various disease-related parameters, viz., reproductive rate, incubation period, transmission rate (TR), and time to hospitalization (TSOH).	SEIR
De La Sen et al. [71]	Study the effect of partial and total quarantine of both infectious and susceptible populations without the inclusion of demography and mortality on the transmission rate of COVID-19.	SIR
Abbasi et al. [72]	Study the effect of quarantine on the infection and recovery rates of COVID-19.	SQEIAR
Khanday et al. [73]	Prediction of the number of infected COVID-19 cases-recovered and death cases.	Machine learning and regression models: SVM, ES, LR, and LASSO
Mojjada et al. [74]	Modeling the infection and deaths for COVID-19 spread.	SIR, RF
Sen and Sen [75]	Modeling the dynamics of COVID-19 transmission in terms of infection rates.	SIR
Goo et al. [76]	Prediction of the number of future infections and mortality rates due to COVID-19.	Hybrid: SEIR, Poisson model, GBA, linear local regression, and negative binomial (NB)
Bernal et al. [77]	Study the effect of Pfizer-BioNTech and Oxford-AstraZeneca on infection, mortality, and alpha (B.1.1.7) variant.	Experimental case study
Tang et al. [78]	Study the effect of Moderna and Pfizer-BioNTech on infection, mortality, and delta (B.1.617.2) variant.	Case study
Bernal et al. [79]	Study the effect of Pfizer-BioNTech and Oxford-AstraZeneca on alpha (B.1.1.7) variant and delta (B.1.617.2) COVID-19 variant.	Experimental case study
Pouwels et al. [80]	Study the effect of Pfizer-BioNTech, Oxford-AstraZeneca, and Moderna on delta (B.1.617.2) COVID-19 variant.	Experimental case study
Mlcochova et al. [81]	Study the effect of Moderna and Oxford-AstraZeneca on infection, mortality, alpha (B.1.1.7), and delta (B.1.617.2) variant.	Bayesian model

**Table 6:** Quality Evaluation Metrics used by the selected articles.

Article Id	Model/algorithm	Reported Quality Evaluation Metric (QEM)
A1	Basic SIR model	CFR = 2.4, training cohort = 0.834, validation cohort = 0.804
A2	SIR model	CFR = 4.6, training cohort = 0.91, validation cohort = 0.86
A3	SIER model	Sensitivity analysis: R0 = 2.7, 95% CI
A4	SIR model	Sensitivity analysis: R0 = 3.1, 95% CI
A5	SIR model	Sensitivity analysis: R0 = 4.3, 95% CI
A6	SIR model	95% CI, prediction cohort = 0.88, validation cohort = 0.831
A7	SVM	Accuracy = 97.5%, specificity = 99.7%, sensitivity = 95.8%
A8	Machine learning models: SVM, RF, LR, and GBA models	SVM: AUC = 0.851, sensitivity = 0.677, specificity = 0.850, F1 score = 0.724, Brier score = 0.160, PPV = 0.778 RF: AUC = 0.851, sensitivity = 0.677, specificity = 0.850, F1 score = 0.724, Brier score = 0.161, PPV = 0.778 LR: AUC = 0.893, sensitivity = 0.742, specificity = 0.825, F1 score = 0.754, Brier score = 0.161, PPV = 0.767 GBA: AUC = 0.842, sensitivity = 0.806, specificity = 0.800, F1 score = 0.781, Brier score = 0.171, PPV = 0.758
A9	DT	AUC = 0.87, sensitivity = 0.807, specificity = 0.801
A10	SIR model	95% CI, training cohort = 0.718, validation cohort = 0.70
A11	Machine learning models: SVM, RF, GBT, LR, and DT models	SVM: AUC = 0.811, sensitivity = 0.650, specificity = 0.880, F1 score = 0.714, Brier score = 0.158 RF: AUC = 0.811, sensitivity = 0.650, specificity = 0.880, F1 score = 0.710, Brier score = 0.156 LR: AUC = 0.831, sensitivity = 0.702, specificity = 0.785, F1 score = 0.730, Brier score = 0.162 GBA: AUC = 0.831, sensitivity = 0.830, specificity = 0.750, F1 score = 0.751, Brier score = 0.131
A12	SIER	R0 = 7.1, prediction cohort = 0.78, testing cohort = 0.73
A13	SIER	R0 = 3.6, prediction cohort = 0.81, testing cohort = 0.78
A14	Machine learning and ensemble models: SVM, LR, RF, AdaBoost, and XGBoost	SVM: AUC = 0.80, sensitivity = 0.680, specificity = 0.890 RF: AUC = 0.80, sensitivity = 0.680, specificity = 0.890 LR: AUC = 0.811, sensitivity = 0.712, specificity = 0.792 AdaBoost: AUC = 0.851, sensitivity = 0.711, specificity = 0.771 XGBoost: AUC = 0.852, sensitivity = 0.721, specificity = 0.780
A15	SIR model	R0 = 2.8, training cohort = 0.88, testing cohort = 0.79
A16	SIER	R0 = 2.3, 95% CI, training cohort = 0.77, testing cohort = 0.78
A17	SIR model	U.K.: R0 = 2.25, training cohort = 0.83, testing cohort = 0.78 Italy: R0 = 2.75, training cohort = 0.85, testing cohort = 0.76
A18	SIIR model: incorporation of I compartment for modeling asymptomatic infections	95% CI
A19	SIER	95% CI, training cohort = 0.85, validation cohort = 0.81
A20	SIRD model	R0 = 2.3, Rt = 2.7, training cohort = 0.84, validation cohort = 0.81
A21	SIRD	R0 = 2.6, prediction cohort = 0.89, validation cohort = 0.85
A22	SIER	Rajasthan: R0 = 4.2, 95% CI Maharashta: R0 = 2.3, 95% CI Gujarat: R0 = 2.7, 95% CI Delhi: R0 = 2.3, 95% CI
A23	SIER	Maharashta: R0 = 4.3, 95% CI Tamil Nadu: R0 = 2.9, 95% CI Delhi: R0 = 3.1, 95% CI
A24	SIER	95% CI, training cohort = 0.714, validation cohort = 0.70
A25	SIR	95% CI, prediction cohort = 0.651, testing cohort = 0.632
A26	SIR	95% CI, prediction cohort = 0.68, testing cohort = 0.63
A27	SIR	95%CI, training cohort = 0.73, testing cohort = 0.70
A28	SEIR	95% CI
A29	SEIR	Beijing: R0 = 4.5 Henan: R0 = 4.3
A30	SIR model	New York: Rt = 4.4, 95% CI Michigan: Rt = 4.5, 95% CI
A31	Logistic growth curve model and time interrupted regression model	R0 = 3.8, 95% CI
A32	Hybrid: SEIR and SVM	Sensitivity analysis: Italy: R0 = 4.5, 95% CI U.K.: R0 = 5.3, 95% CI
A33	Holt model, ARIMA, TBATS, and cubic smoothing spline model	ARIMA: MAPE = 5.2%, MAE = 5.3, AIC = 5.5 TBATS: MAPE = 8.1%, MAE = 7.9, AIC = 7.8 Spline: MAPE = 5.9%, MAE = 5.7, AIC = 5.4 Holt: MAPE = 6.8%, MAE = 6.6, AIC = 6.7
A34	SIR model	R0 = 2.8, 95% CI
A35	SEIR	R0 = 4.3,95% CI, prediction cohort = 0.83, validation cohort = 0.81
A36	SEIR with ARIMA corrections	95% CI, prediction cohort = 0.73, validation cohort = 0.70
A37	SIR	UIR = 20%, IFR = 0.61, TR = 0.03%, 95% CI
A38	SEIR	First wave: R0 = 6.49, 95% CI Second wave: R0 = 6.2, 95% CI Third wave: R0 = 4, 95% CI
A39	SEIR	R0 = 3.5, 95% CI, training cohort = 0.89, validation cohort = 0.83
A40	SIR	95% CI, prediction cohort = 0.82, validation cohort = 0.78
A41	SQEIAR	China: prediction cohort = 0.782, validation cohort = 0.77 Spain: prediction cohort = 0.772, validation cohort = 0.745
A42	Machine learning and regression models: SVM, DT, LR, RF, and AdaBoost	SVM: precision = 0.82, recall = 0.91, F1 score = 0.86, accuracy = 90.6% LR: precision = 0.94, recall = 0.96, F1 score = 0.95, accuracy = 96.2% DT: precision = 0.92, recall = 0.92, F1 score = 0.92, accuracy = 92.5%, AdaBoost: precision = 0.85, recall = 0.91, F1 score = 0.88, accuracy = 90.6% RF: precision = 0.93, recall = 0.94, F1 score = 0.93, accuracy = 94.3%
A43	SIR, RF	SIR: R0 = 3.8, 95% CI RF: sensitivity = 0.93, recall = 0.91
A44	SIR	95% CI, prediction cohort = 0.86, validation cohort = 0.84
A45	Hybrid: SEIR, GBA, and linear local regression	SEIR:95% CI GBA: AUC = 0.811, sensitivity = 0.650, specificity = 0.880, F1 score = 0.710, Brier score = 0.156 LLR: AUC = 0.831, sensitivity = 0.702, specificity = 0.785, F1 score = 0.730, Brier score = 0.162, RMSE: LMST = 30.12
A46	Experimental case study	95% CI, training cohort = 0.79, validation cohort = 0.80
A47	Case study	95% CI, prediction cohort = 0.93, validation cohort = 0.86
A48	Experimental case study	95% CI, training cohort = 0.718, validation cohort = 0.70
A49	Experimental case study	95% CI, prediction cohort = 0.86, validation cohort = 0.84
A50	Bayesian model	95% CI, AUC = 0.77, AIC = 0.73

**Table 7:** Identified key-disease related parameters and control measures for SARS-COVID-19.

Article Id	Estimated/evaluated epidemiological parameters	Control measures incorporated
A1	CFR	—
A2	CFR	—
A3	Reproductive rate (R0), travel considerations	—
A4	Reproductive rate (R0), CFR	Quarantine
A5	Reproductive rate (R0)	—
A6	Infection and death rates	Lockdown
A7	Infection and death rates	—
A8	Infection and death rates	Testing and tracing application
A9	Infection and death rates	—
A10	Infection and death rates	Quarantine
A11	Infection and death rates	—
A12	Reproductive rate (R0), infection and death rates	Lockdown
A13	Reproductive rate (R0)	—
A14	Reproductive rate (R0)	—
A15	Reproductive rate (R0) infection and death rates	Quarantine
A16	Reproductive rate (R0) infection and death rates	Lockdown
A17	Reproductive rate (R0), herd immunity	Lockdown
A18	HIT	—
A19	Asymptomatic infection rate	Quarantine, contact rate, lockdown
A20	Infection and death rates	Quarantine and lockdown
A21	CFR, reproductive rate (R0)	Quarantine
A22	Contact rate, reproductive rate (R0)	Lockdown
A23	Reproductive rate (R0)	Quarantine and lockdown
A24	Asymptomatic infection rate, transmission rate	—
A25	Transmission rate	Quarantine, social distancing
A26	Infection and death rate	Contact rate
A27	Transmission rate	—
A28	Infection and death rate	Social distancing, undetected infection rate, testing and tracing apps
A29	Reproductive rate (R0)	Quarantine
A30	Infection and death rate	Lockdown, testing and tracing apps
A31	Infection and death rate	Lockdown, quarantine
A32	Reproductive rate (R0)	Lockdown
A33	Reproductive rate (R0)	Social distancing, contact rate
A34	Reproductive rate (R0)	Social distancing, contact rate
A35	Reproductive rate (R0)	Quarantine, social distancing,
A36	Infection and death rate	Quarantine, unidentified infection rate
A37	IFR, TR	Lockdown, quarantine, undetected infection rate
A38	Reproductive rate (R0), infection and death rate	—
A39	Reproductive rate (R0), TSOH	Social distancing, hospitalization, quarantine, travel restrictions, contact tracing
A40	Transmission rate	Quarantine, hospitalization
A41	Asymptomatic infection rate	Quarantine, travel restrictions, undetected infection rate
A42	Infection and death rates	Lockdown
A43	Reproductive rate (R0), infection and death rates	Quarantine
A44	Infection and death rates	Quarantine, lockdown
A45	Infection and death rates	Quarantine
A46	Effectiveness of Pfizer-BioNTech and Oxford-AstraZeneca on alpha (B.1.1.7) variant	—
A47	Effect of Moderna and Pfizer-BioNTech on delta (B.1.617.2) variant	—
A48	Effectiveness of Pfizer-BioNTech and Oxford-AstraZeneca on alpha (B.1.1.7) variant and delta (B.1.617.2) COVID-19 variant	—
A49	Effect of Pfizer-BioNTech, Oxford-AstraZeneca, and Moderna on delta (B.1.617.2) COVID-19 variant	—
A50	Study the effect of Moderna and Oxford-AstraZeneca on infection, mortality, alpha (B.1.1.7), and delta (B.1.617.2) variant	—

## Data Availability

Publicly available datasets were analyzed in this study. These datasets can be found at https://github.com/CSSEGISandData/COVID-19. Detailed links are given in references.
